# Ameliorative Potential of Resveratrol in Dry Eye Disease by Restoring Mitochondrial Function

**DOI:** 10.1155/2022/1013444

**Published:** 2022-05-26

**Authors:** Jingyao Chen, Weijia Zhang, Yixin Zheng, Yanze Xu

**Affiliations:** Department of Ophthalmology, Yan An Hospital Affiliated to Kunming Medical University, Kunming, China

## Abstract

**Methods:**

The mitochondrial dysfunction of HCE-2 human corneal epithelial cells was induced by high osmotic pressure exposure and treated with resveratrol (50 *μ*M). Western blotting was used to detect the expression of the antioxidant proteins SOD2, GPx, and SIRT1, and flow cytometry was used to detect cell apoptosis and ROS production. The DED mouse model was induced by 0.2% benzalkonium chloride (BAC) and treated with resveratrol. The tear yield was measured by the phenol cotton thread test, the density of cup cells in the conjunctiva was measured by periodic acid-Schiff (PAS) staining, and the expression levels of SIRT1, GPx, and SOD2 in lacrimal glands were detected by Western blotting.

**Results:**

In hypertonic conditions, the apoptosis of HCE-2 cells increased, the expression of the antioxidant proteins SOD2 and GPx decreased, ROS production increased, and the expression of SIRT1 protein, an essential regulator of mitochondrial function, was downregulated. Treatment with resveratrol reversed the mitochondrial dysfunction mediated by high osmotic pressure. In the DED mouse model, resveratrol treatment promoted tear production and goblet cell number in DED mice, decreased corneal fluorescein staining, upregulated SIRT1 expression, and induced SOD2 and GPx expression in DED mice.

**Conclusion:**

Resveratrol alleviates mitochondrial dysfunction by promoting SIRT1 expression, thus reducing ocular surface injury in mice with dry eye. This study suggests a new path against DED.

## 1. Introduction

 DED is a prevalent ocular surface disorder caused by inadequate production of tears and excessive tear evaporation. Of note, the prevalence of DED in the world population ranges from 6 to 34%, and the prevalence of DED is higher in the aging population [1]. Thus, effective therapeutic strategies are urgently needed for remitting DED.

Emerging evidence indicates that mitochondrial dysfunction is responsible for pathological processes, including but not limited to neurodegenerative disease [2], cancer [3], and DED [4]. Studies have shown that mitochondrial function is a crucial component in the progression of DED. For example, DDIT4 knockdown restores mitochondrial function under hyperosmolarity and preserves the viability of human corneal epithelial cells [5]. Moreover, the modulation of mitochondrial homeostasis is related to the outcome of DED [6]. Recent studies suggest that antioxidant administration may restore mitochondria. Resveratrol (3,5,4′-trihydroxy-trans-stilbene), a natural plant product, has been reported to have antioxidant effects and maintain mitochondrial function [7, 8]. The protective role of resveratrol in mitochondrial dysfunction-related diseases, such as cardiac diseases [9], hypoxic ischemic injury [10], and neurodegenerative disorders [11], has been well established. It is worth noting that the function of resveratrol in protecting the ocular surface in experimental DED has been reported [12]. However, the underlying mechanism by which resveratrol ameliorates DED remains obscure.

Mammalian sirtuin 1 (SIRT1) is an exceedingly conserved NAD(+)-dependent deacetylase that has been reported to be engaged in the regulation of mitochondrial biogenesis [13]. Aberrant expression of SIRT1 leads to mitochondrial dysfunction, thereby enhancing pathological processes [14]. Earlier research revealed that the expression of SIRT1 is decreased in the condition of diabetic dry eye [15], indicating that SIRT1 may function in DED. It is well known that resveratrol is a potent activator of SIRT1 [16]. Currently, the antioxidative effect of resveratrol is achieved by upregulating SIRT1 expression [17]. For instance, resveratrol improves mitochondria and protects against metabolic disease by activating SIRT1 [18]. Resveratrol activates SIRT1 to alleviate cardiac dysfunction through mitochondrial regulation [19]. However, the correlation between resveratrol and SIRT1 in DED is unknown.

Thus, we demonstrate that resveratrol treatment attenuates hyperosmolarity-induced mitochondrial dysfunction in human corneal epithelial cells (HCEpiCs). SIRT1 is reduced in hyperosmolarity-treated HCEpiCs, while resveratrol upregulates SIRT1 expression. Moreover, we found that resveratrol restores mitochondrial function by inducing SIRT1 expression. Consistently, resveratrol ameliorated dry eye symptoms in the DED mouse model. Thus, our results establish a novel mechanism by which resveratrol attenuates DED by facilitating SIRT1 expression.

## 2. Materials and Methods

### 2.1. Cell Culture and Treatment

Human corneal epithelial cells HCE-2[50.B1] (CRL-11135) were acquired from ATCC (Manassas, VA, USA). Cells were cultured at 37°C in 5% CO_2_ humidity in 10% fetal bovine serum (FBS, Gibco) and 1% v/v penicillin/streptomycin (Gibco) in Dulbecco's modified Eagle's medium (DMEM, Gibco). For the DED cell model, HCEpiCs were treated with 0 or 94 mM NaCl in the medium and treated at isotonic and high osmolarity (312 and 500 mOsM) for 24 h. For resveratrol treatment, HCEpiCs were administered at 50 *μ*M, and the vehicle (alcohol) had a final concentration of 0.5% (nontoxic for cells) [20].

### 2.2. Cell Apoptosis Assay

The apoptosis of the indicated cells was analyzed by an Annexin V-FITC apoptosis detection kit (C1062S, Beyotime). Briefly, cells were collected and resuspended in PBS. After centrifugation, the suspension was discarded, and the cells were resuspended in buffer. Subsequently, 5 *μ*l of Annexin V-FITC and 10 *μ*l of propidium iodide staining solution were added. After incubating at room temperature in the dark for 10–20 minutes, the cells were placed on ice and analyzed by flow cytometry.

### 2.3. Measurement of ROS Levels

The ROS level in the indicated cells was measured by an ROS assay kit (ab113851, Abcam). Briefly, HCEpiCs were stained with DCFDA for 30 minutes at 37°C.

### 2.4. Western Blot

Proteins isolated from HCEpiCs and lacrimal glands were measured by a BCA assay kit (P0012S, Beyotime). Approximately 40 *μ*g of protein was separated by sodium dodecyl sulfate-polyacrylamide gel electrophoresis (SDS-PAGE) and transferred to PVDF membranes (1620177, BioRad). PVDF membranes were blocked in 5% nonfat milk and incubated with the primary antibodies at 4°C overnight. After washing with TBST three times, the membranes were incubated with secondary antibodies. Finally, the bands were measured with an ECL reagent kit (A38555, Thermo Scientific™).

### 2.5. Animal Model and Treatment

Seventy female C57BL/6 mice (Certificate number: SCXK(Dian)K2020-0004) aged 6–8 weeks were purchased from the Animal Center of Kunming Medical University. The mice were instilled with 5 *μ*L of 0.2% BAC (Sigma-Aldrich) solution in both the eyes, twice a day, for 2 consecutive weeks, to induce the mouse DED model [21]. After the successful establishment of the DED model, the mice were randomly divided into 3 groups (15 mice in each group): DED group, DED mice with alcohol administration, and DED mice with resveratrol administration, and the mice without BAC induction were used as the normal control group. Resveratrol (5 *μ*L/eye) was administered 3 times/day in both the eyes for two weeks. Eventually, the mice were euthanized by CO_2_ asphyxiation, and the entire eye tissue, including the conjunctiva and eyeball, was removed for further analysis.

### 2.6. Corneal Fluorescein Staining

1 *μ*L of 1% sodium fluorescein was dropped into the inferior conjunctival sac using a micropipette; then, punctate staining on the corneal surface was evaluated in a blind fashion. Cobalt blue light was used for inspection and photographic recording under a slit-lamp microscope with 0 points for no staining of corneal fluorescein, 1 point for one-quarter staining, 2 points for less than half staining, 3 points for more than half staining, and 4 points for more than half staining [22].

### 2.7. Tear Production

The tear output was analyzed using phenol red cotton threads (Tianjin Jingming) [23]. The phenol red thread was positioned in the lateral canthus of the eye for 60 seconds, and then, thread wetting measurements were recorded.

### 2.8. Periodic Acid-Schiff (PAS) Staining

The eyeball was embedded and sliced into 5 *μ*m thick divisions. Each division was stained with periodic acid-Schiff (PAS) [24]. The goblet cell density was quantified.

### 2.9. Statistical Analysis

All data are expressed as the mean ± SEM. GraphPad software was used to analyze and draw figures. The statistical significance of differences was evaluated by the two-tailed Student's *t*-test or two-way ANOVA. All *p* values were considered statistically significant when values were <0.05.

## 3. Results

### 3.1. Environmental Hyperosmolarity Promotes Mitochondrial Dysfunction in HCEpiCs

To investigate the part of mitochondria in DED, a hyperosmolarity HCEpiCs model was created using 500 mOsM medium, and HCEpiCs exposed to 312 mOsM medium were regarded as controls. As shown in Figure 1(a), after exposure to 500 mOsM medium, the apoptosis of HCEpiCs was increased. The expression levels of the antioxidant proteins SOD2 and GPx were reduced in HCEpiCs under hyperosmolarity (Figure 1(b)). Consistently, hyperosmolarity increased ROS production in HCEpiCs (Figure 1(c)).

### 3.2. Resveratrol Treatment Suppresses Mitochondrial Dysfunction in HCEpiCs

Resveratrol is reported to modulate mitochondrial function in vitro and in vivo. To understand the function of resveratrol in mitochondrial function in HCEpiCs, hyperosmolarity-treated HCEpiCs were administered 50 *μ*m of resveratrol. The apoptosis of HCEpiCs was reduced by resveratrol treatment (Figure 2(a)). Resveratrol administration promoted SOD2 and GPx expression (Figure 2(b)); in contrast, ROS production was reduced (Figure 2(c)).

### 3.3. Resveratrol Upregulates SIRT1 Expression in HCEpiCs

Previous studies suggested that SIRT1 contributed to mitochondrial function maintenance [25]. SIRT1 is involved in resveratrol-mediated mitochondrial regulation [19, 26]. Here, we showed that SIRT1 was suppressed in HCEpiCs under hyperosmolarity (Figure 3(a)). We examined the effects of resveratrol on SIRT1 and found that the expression of SIRT1 was recovered with resveratrol treatment (Figure 3(b)).

We next asked whether SIRT1 was responsible for resveratrol-mediated mitochondrial regulation in HCEpiCs. To test this hypothesis, we introduced the SIRT1 inhibitor EX527. Treatment with EX527 counteracted the inhibitory effect of resveratrol on HCEpiCs apoptosis (Figure 3(c)) and SOD2 and GPx expression (Figure 3(d)). We also observed that EX527 eliminated part of the inhibitory effect of resveratrol on ROS production (Figure 3(e)).

### 3.4. Resveratrol Ameliorates DED Syndrome in Vivo via SIRT1

Next, a DED mouse model induced by BAC ammonium chloride was used to determine the role of resveratrol in DED progression. Tear output was measured by the phenol red cotton thread test, which indicated that resveratrol-treated DED mice experienced more tear production than alcohol-treated DED mice and DED mice (Figure 4(a)). Corneal fluorescein staining was decreased in resveratrol-treated mice (Figure 4(b)). Moreover, the number of goblet cells was increased with resveratrol administration (Figure 4(c)). These data indicated that resveratrol attenuates DED progression.

We then detected SIRT1 expression in lacrimal glands and found that SIRT1 was inhibited in DED mice and alcohol-treated DED mice, while resveratrol upregulated SIRT1 expression (Figure 4(d)). Moreover, resveratrol administration induced SOD2 and GPx expression in the DED mouse model (Figure 4(e)).

## 4. Discussion

In the current research, we demonstrated that hyperosmolarity induces apoptosis and mitochondrial dysfunction in HCEpiCs, while resveratrol restores the mitochondrial function of HCEpiCs under hyperosmolarity. Decreased expression of SIRT1 could be observed in HCEpiCs with hyperosmolarity culturing. Importantly, our results further demonstrated that SIRT1 is responsible for resveratrol-mediated mitochondrial restoration. Consistently, by establishing a DED mouse model, we found that resveratrol prevents DED syndrome. Thus, our data extended the role of resveratrol and illustrated the underlying mechanism of resveratrol in ameliorating DED.

DED is a multifactorial disease and is closely related to mitochondrial function. In diabetic mice, Qu et al. [27] demonstrated that hyperglycemia-induced mitochondrial bioenergetic inadequacy of the lacrimal gland ameliorates early onset of dry eye. Bogdan et al. [28] proposed that insulin-like growth factor binding protein-3 (IGFBP-3) is involved in hyperosmolar stress responses in the corneal epithelium by modulating mitochondrial function. Hyperosmolarity can increase ROS and apoptosis of HCEpiCs (Figure 1), and our results confirm this. Since antioxidants are one of the most common factors for restoring mitochondrial function and could prevent mitochondrial-associated pathology [29], we focused on resveratrol and set out to determine the role of resveratrol in DED development. Resveratrol, a common antioxidant, contributes to mitochondrial function maintenance. Kang et al. [30] showed that resveratrol protects neural cells from injury via regulation of mitochondrial biogenesis and mitophagy. In C6 astrocytes, Bobermin et al. [31] demonstrated that resveratrol prevents an increase in ROS production, a reduction in mitochondrial membrane potential (ΔΨ), and bioenergetic insufficiency caused by ammonia. Importantly, several studies have indicated that resveratrol prevents DED syndrome [12, 32]. However, whether resveratrol attenuates DED development by regulating mitochondria remains unknown. Here, we found that hyperosmolarity culturing reduces the expression of the antioxidant proteins SOD2 and GPx and induces ROS levels. Resveratrol administration inhibits HCEpiCs apoptosis, increases SOD2 and GPx expression, and decreases ROS levels. Moreover, resveratrol attenuates DED syndrome and increases SOD2 and GPx expression in a DED mouse model. These results suggest that resveratrol may reduce oxidative stress and HCEpiCs apoptosis by maintaining mitochondrial function.

SIRT1 contributes to the function and biogenesis of mitochondria [33]. Of note, Samadi et al. [34] described that SIRT1 expression is suppressed in a diabetic dry eye model. Here, we also observed decreased expression of SIRT1 in HCEpiCs from a hyperosmolarity culture and DED mouse model, which was accompanied by increased levels of oxidative stress, apoptosis, or dry eye syndrome. In addition, resveratrol was previously shown to be critical in SIRT1 activation [35]. In the next experiment, we demonstrated that resveratrol treatment reversed SIRT1 expression in HCEpiCs under hyperosmolarity and DED in mice, while the SIRT1 inhibitor EX527 rescued the inhibitory effect of resveratrol on mitochondrial dysfunction in HCEpiCs. This finding suggests that resveratrol ameliorates mitochondrial dysfunction via SIRT1.

It was proposed in early studies that the antioxidant resveratrol is critical in preventing DED syndrome, but the mechanism remains unclear. Our results demonstrate that resveratrol can restore mitochondrial function in HCEpiCs and inhibit HCEpiCs apoptosis. Furthermore, our findings indicate that SIRT1 is the major effector in resveratrol-regulated DED development. Therefore, our results show that resveratrol/SIRT1 plays a significant role in DED development, which is beneficial to DED therapy.

## 5. Conclusion

In summary, we found that resveratrol reversed hyperosmolarity-mediated mitochondrial dysfunction in HCEpiCs, and we demonstrated that resveratrol alleviated mitochondrial dysfunction by promoting SIRT1 expression. At the same time, it has been proven in animal experiments that resveratrol can reduce ocular surface damage in a mouse model of DED. Finally, resveratrol improved the effect of DED by restoring mitochondrial function, and this study provides new ideas for the treatment of DED.

## Figures and Tables

**Figure 1:** Environmental hyperosmolarity promotes mitochondrial dysfunction in HCEpiCs. (a) Apoptosis of HCEpiCs under iso and hyperosmolarities (312 and 500 mOsM) determined by flow cytometry. (b) The expression levels of the antioxidant proteins SOD2 and GPx measured by Western blotting. (c) ROS production under iso- and hyper-osmolarities determined by flow cytometry. *n* = 3. ^∗^*P* < 0.05 and ^∗∗∗^*P* < 0.001.

**Figure 2:** Resveratrol treatment suppresses mitochondrial dysfunction in HCEpiCs. (a) Apoptosis of HCEpiCs under hyperosmolarity (500 mOsM) with resveratrol treatment determined by flow cytometry. (b) The expression levels of the antioxidant proteins SOD2 and GPx measured by Western blotting. (c) ROS production in HCEpiCs under hyperosmolar conditions with resveratrol treatment determined by flow cytometry. *n* = 3. ^*∗*^*P* < 0.05, ^*∗∗*^*P* < 0.01, ^∗∗∗^*P* < 0.01.

**Figure 3:** Resveratrol upregulates SIRT1 expression in HCEpiCs. (a) Expression of SIRT1 in HCEpiCs under iso- and hyper-osmolarities (312 and 500 mOsM) detected by Western blotting. (b) Expression of SIRT1 in HCEpiCs under hyperosmolarity (500 mOsM) with resveratrol treatment determined by Western blotting. (c) Apoptosis of HCEpiCs under hyperosmolar conditions treated with resveratrol and/or the SIRT1 inhibitor EX527 determined by flow cytometry. (d) Expression of SIRT1, GPx, and SOD2 in HCEpiCs under hyperosmolarity with resveratrol and/or SIRT1 inhibitor EX527 treatment measured by Western blotting. (e) ROS production in HCEpiCs under hyperosmolar conditions treated with resveratrol and/or the SIRT1 inhibitor EX527 measured by flow cytometry. *n* = 3. ^*∗*^*P* < 0.05, ^*∗∗*^*P* < 0.01, ^∗∗∗^*P* < 0.001.

**Figure 4:** Resveratrol ameliorates DED syndrome in vivo via SIRT1. (a) The tear production in control mice, DED mice, DED mice treated with alcohol, or DED mice treated with resveratrol measured by the phenol red cotton thread test. (b) Corneal fluorescein staining in control mice, DED mice, DED mice with alcohol treatment, and DED mice treated with resveratrol. (c) Goblet cell density in the conjunctival epithelial layer measured by periodic acid-Schiff (PAS) staining. (d) Expression of SIRT1 in lacrimal glands determined by Western blotting. (e) Expression of GPx and SOD2 in lacrimal glands determined by Western blotting. *n* = 3. ^*∗*^*P* < 0.05, ^*∗∗*^*P* < 0.01, ^∗∗∗^*P* < 0.001.

## Data Availability

The datasets generated during and/or analyzed during the current study are available from the corresponding author upon request.
